The article "The emerging roles and functions of circular RNAs and their generation" was published in 2019. Journal: J Biomed Sci.

# The emerging roles and functions of circular RNAs and their generation

**DOI:** 10.1186/s12929-019-0523-z

**Published:** 2019-04-25

**Authors:** Chun-Ying Yu, Hung-Chih Kuo

**Affiliations:** 1 Institute of Cellular and Organismic Biology, Academia Sinica, No. 128, Sec. 2, Academia Road, Nankang, Taipei, 11529 Taiwan; 2 Department of Biomedical Sciences, National Chung Cheng University, Chiayi, Taiwan; 3 Graduate Institute of Medical Genomics and Proteomics, College of Medicine, National Taiwan University, Taipei, Taiwan

**Keywords:** Circular RNAs (circRNAs), Splicing factor, Micro RNAs (miRNAs), Long non-coding RNAs (lncRNAs)

## Abstract

Circular RNAs (circRNAs) are closed long non-coding RNAs, in which the 5’ and 3’ termini are covalently linked by back-splicing of exons from a single pre-mRNA. Emerging evidence indicates that circRNAs are broadly expressed in mammalian cells and show cell type- or tissue-specific expression patterns. Importantly, circRNAs have been shown to participate in regulating various biological processes. Functionally, circRNAs can influence cellular physiology through various molecular mechanisms, such as serving as a decoy for microRNAs or RNA-binding proteins to modulate gene expression or translation of regulatory proteins. The biogenesis of circRNAs is known to be tightly regulated by *cis-* (intronic complementary sequences) and/or trans-factors (splicing factors) that constitute a cell- and context-dependent regulatory layer in the control of gene expression. However, our understanding of the regulation and function of circRNAs is still limited. In this review, we summarize the current progress in elucidating the functional roles, mechanisms and biogenesis of circRNAs. We also discuss the relationship between regulation and formation of circRNAs.

## Background

As most eukaryotic genes are interrupted by non-informational introns, nascent RNA transcripts typically undergo splicing to remove introns, after which the exons are fused colinearly to form mature linear RNA transcripts (Fig. 1). Splicing is a highly regulated process, which may generate multiple mature RNA isoforms from a given gene, and these isoforms may exhibit different functions, cellular locations or regulatory roles [1]. Over 95% of human genes have alternatively spliced isoforms [2], the expression of which is determined by both trans-regulatory factors and *cis*-regulatory elements, including splicing factors and their binding motifs.

**Fig. 1:** Back-splicing and canonical splicing of a single pre-mRNA. (**a**) The single pre-mRNA can be back-spliced with the 5’ terminus of upstream exon 2 ligated to the 3′ terminus of downstream exon 3 to generate a circRNAs. (**b**) Otherwise, the exons of the pre-mRNA can be joined colinearly by canonical splicing to form mRNAs or lncRNAs

Circular RNAs (circRNAs) are generated by a specific type of splicing called back-splicing, wherein the 5’ terminus of a pre-mRNA upstream exon is non-colinearly spliced with the 3’ terminus of a downstream exon (Fig. 1). CircRNAs are predominantly found in the cytoplasm, and the lack of a 5’ cap and 3’ tail make the circular molecules more resistant to RNase degradation compared to their linear cognates [3]. The existence of mammalian circRNAs was first reported in 1979 by Hsu, who observed the molecules in the cytoplasm of HeLa and other mammalian cells by electron microscopy [4]. However, due to technical limitations, only a few specific circRNAs were identified throughout the next two decades, and the potential functions of circRNAs remained unclear [5–9]. With the development of next generation sequencing, alongside the publication of complete genome sequences and the advance of bioinformatics technology, researchers have discovered that the expression of circRNAs in mammals is often conserved across species, and shows tissue and cell specificity. The expression level of some circRNAs can be higher than the linear cognates [10–14].

Importantly, Memczak et al. and Hansen et al. first demonstrated that the circular isoform of human antisense to cerebellar degeneration-related protein 1 RNA (*CDR1as*) is functional in neural development, and this striking observation launched the nascent field of circRNA research [15, 16]. The number of published circRNA studies has grown exponentially in the following years, making circRNAs some of the most notable molecules in RNA biology. Several databases (e.g., circBase, circNet, Circ2Traits, exoRBase, and CSCD) have been created to curate circRNAs from different species and provide further information about association with diseases, cellular locations and other non-coding RNAs. The availability of this information speeds up the exploration of circRNA functions and underlying mechanisms by which circRNAs exert functions [17–22].

Although most circRNAs are spliced from protein coding pre-mRNAs, circRNAs are usually categorized as long non-coding RNAs (lncRNAs). Similar to other lncRNAs, circRNAs can serve as RNA or protein decoys to regulate gene expression. The most well-known type of circRNA interaction is with microRNAs (miRNAs). Individual circRNAs can harbor multiple miRNA binding sites to act as a “sponge” and inhibit activity of one or multiple miRNAs. CircRNAs also form complexes with proteins to regulate the cell cycle [23] or translation [24], or to serve as intercellular signaling molecules in released exosomes [25, 26]. Interestingly, some circRNAs may encode functional peptides, as demonstrated in recent work showing that circRNAs were able to be translated in vitro and in vivo [27–30].

CircRNA formation competes with formation of linear cognates, indicating that the canonical spliceosome has some involvement in back-splicing [31, 32]. Short intronic repeats or Alu elements promote circRNA formation in cis [33–35], whereas RNA binding proteins (e.g., splicing factors) play important roles in regulating circRNA formation in trans [32, 36–38]. Despite many exciting advances in circRNA biology, the number and identities of molecules involved in circRNA biogenesis and how regulatory networks control circRNA function remained largely unclear. In this review, we summarize the known functions of circRNAs in mammalian cells and the mechanisms by which circRNAs exert these functions. We also survey the factors that regulate circRNA formation and discuss the relationship between function and formation of circRNAs.

### CircRNAs regulate cell proliferation

Accurate and precise control of the cell cycle is important during normal cellular responses to environmental cues. Dysregulation of the cell cycle in neural stem cells may cause megalencephaly or microcephaly [39], while a lack of cell cycle control in somatic cells can promote cancer progression [40]. A growing number of circRNAs have been reported to regulate proliferation through effects on signaling pathways, transcription factors and cell cycle checkpoint regulators. Two major pathways that regulate cell proliferation and are affected by circRNAs include MAPK/ERK and PI3K/AKT. In the MAPK/ERK pathway, growth factors (e.g., FGF) bind to receptor tyrosine kinases (e.g., FGFR), which then phosphorylate MAPK to activate ERK and promote cell proliferation. *CDR1as* and *circHIPK3* were shown to promote EGFR receptor expression in colorectal cancer (CRC) and esophageal squamous cell carcinoma (ESCC) [41, 42], while *circWDR77* enhanced FGF2 ligand expression in vascular smooth muscle cells [43](Fig. 2a). In the PI3K/AKT pathway, ligands (e.g., insulin) bind to receptor tyrosine kinases, which activate PI3K to phosphorylate AKT and promote cell proliferation. In hepatocellular carcinoma (HCC) and glioblastoma, *CDR1as* and *circNT5E* were found to promote cell proliferation by increasing PI3K expression [44, 45] (Fig. 2b). CircRNAs also regulate the WNT/β-catenin pathway to promote proliferation. For example, knockdown of *circHIPK3* was shown to decrease WNT2 ligand and FZD4 receptor expression, which decreased the level of nuclear β-catenin and hampered retinal endothelial cell proliferation [46]. Moreover, *circZFR* potentiated β-catenin expression in HCC and promoted proliferation [47] (Fig. 2c). In addition, *circHIPK3* can promote proliferation in human cell lines, probably through upregulation of IL6R expression [48]. Transcription factors and cell cycle checkpoints are also found to be targets of circRNA regulation. For instance, disruption of *circTCF25* and *circRNA_100290* in cancer cells downregulates CDK6 expression, affecting the proliferation of bladder cancer and osteosarcoma cells [49, 50] (Fig. 2d). Moreover, circRNA *hsa_circ_0008039* is reported to increase E2F3 expression, inducing S-phase transition and promoting proliferation of breast cancer cells [51] (Fig. 2d). On the other hand, circRNAs may also inhibit cell proliferation. Ectopic expression of *circITCH* and *circZFR* upregulates PTEN expression, which inhibits proliferation of bladder cancer and HCC cells [52, 53] (Fig. 2d). Furthermore, *circITCH* promotes ITCH and CBL expression, which inhibits cell proliferation by downregulating the WNT/β-catenin pathway [54, 55] (Fig. 2c). Similarly, *hsa_circ_0002052* induces APC2 expression, which promotes β-catenin degradation to inhibit osteosarcoma cells proliferation [56] (Fig. 2c). In another example, *circFOXO3* is shown to interact with and sequester P21 and CDK2 in the cytoplasm, attenuating cell cycle progression [23] (Fig. 2d). Together, these reports demonstrate that circRNAs can regulate cell proliferation through a variety of different mechanisms.

**Fig. 2:** CircRNA regulates cell proliferation. CircRNA regulates cell proliferation through multiple factors, including (**a**) FGF2 and EGFR in MAPK/ERK pathway, (**b**) PI3K in PI3K/AKT pathway, (**c**) WNT2, FZD4, ITCH, CBL, APC2, and β-catenin in WNT/β -catenin pathway, and (**d**) CDK6, E2F3, PTEN, P21 and CDK2 that regulate cell cycle. CircRNAs promote or inhibit cells proliferation are labeled by black and red, respectively

### CircRNAs regulate epithelial-mesenchymal transition (EMT) and cancer progression

EMT is highly regulated during development to ensure correct localization of differentiated cells at the proper times. The improper activation of EMT is frequently found in the early stages of cancer progression and causes cancer cell migration and invasion. EMT is mainly induced by TGF-β family ligands, which stimulate the phosphorylation and nuclear translocation of R-SMADs and co-SMADs to activate SNAI, bHLH and ZEB transcription factors [57]. Accumulating evidence suggests that circRNAs contribute to cancer progression by regulating the EMT process. *circMYLK* was found to act on the TGF-β signaling pathway by increasing TRAF4 expression in PC-a cells to attenuate degradation of the TGF-β receptor and promote EMT [58]. *circRNA_0084043* also promoted EMT by upregulating SNAI expression in melanoma cells [59]. Similarly, *circIRAK3, circNASP, circMAN2B2* and *circSHKBP1* respectively promoted FOXC1, FOXF1, FOXK1 and FOXP1 expression, all of which upregulated SNAI expression in cancer cells [60–63]. CircRNAs have also been shown to inhibit EMT. For example, *circSMAD2* upregulated TRIM33, which trapped SMAD4 to block the TGF-β signaling cascade in HCC cells [64]. Additionally, disruption of *circFOXO3* decreased FOXO3 expression, which promoted EMT in non-small-cell lung carcinoma (NSCLC) [65]. These results are summarized in Fig. 3.

**Fig. 3:** CircRNA regulates EMT and cancer progression. CircRNA regulates EMT and cancer progression through multiple factors, including TRAF4, TRIM33, SNAI, FOXC1, FOXF1, FOXK1, FOXO3 and FOXP1 in TGF- β pathway. CircRNAs promote or inhibit EMT are labeled by black and red, respectively

### CircRNAs regulate pluripotency and early lineage differentiation

Pluripotent stem cells, including embryonic stem cells (ESCs) and induced pluripotent stem cells (iPSCs), are able to differentiate into many cell types in our body or in culture. In human ESCs and iPSCs, disruption of *circBIRC6* and *circCOROC1* negatively affects pluripotency maintenance, whereas expression of *circBIRC6* and *circCORO1C* promotes pluripotency reprogramming of iPSCs. Further exploration of the regulatory mechanisms reveals that *circBIRC6* inhibits the activity of miR-34a and miR-145, preventing downregulation of pluripotency transcription factors NANOG, OCT4 and SOX2 [36]. These results suggest that circRNAs play roles in pluripotency maintenance and differentiation. In line with this finding, a recent study of global circRNA expression during human ESCs differentiation showed that *circRMST* and *circFIRRE* are enriched in differentiated hESCs, suggesting that certain circRNAs are associated with ESC differentiation [66]. Further, circRNAs are also involved in somatic stem cell differentiation. For example, *CDR1as* is shown to regulate neural development in zebrafish and osteoblastic differentiation of periodontal ligament stem cells (PDLSC), while ectopic expression of *circFGFR4*, *circSVIL* and *circZNF609* induce myoblast differentiation [15, 67–71]. Interestingly, *circZNF609* may also promote myoblast differentiation through the actions of an encoded small peptide [27].

### Other circRNA functions

CircRNAs have also been shown to also regulate unique functions of specialized cells. For example, *SRY* is a well-known sex determining gene for testis development, which encodes both linear and circular RNAs [5, 72]. In addition to being translated into SRY protein, the RNA product of *SRY* may also serve as a sponge for miR-138 [15]. Another known example of circRNA function in specialized cells is β-cells in pancreatic islets, which produces and secretes insulin. Both *CDR1as* and *circHIPK3* were found to promote insulin secretion from β-cells [73, 74]. In the immune system, *circZC3H4* and *circHECTD1* can promote the activation of alveolar macrophages, which stimulates fibroblast proliferation and migration [75, 76]. In the nervous system, disruption of *circHIPK2* and *circHECTD1* inhibits astrocyte activation, which may be beneficial during stroke recovery [77, 78]. Few circRNAs were reported to regulate apoptosis. In two contrasting examples, *hsa_circ_0043256* induces apoptosis by increasing ITCH in NSCLC cells, but *circGRB10* inhibits apoptosis by increasing ERBB2 in nucleus pulposus (NP) cells [79, 80]. Finally, circRNAs also play important roles in several human diseases. It was previously reported that *circANRIL* interacts with PES1 to regulate rRNA maturation and promotes the development of atherosclerosis [81]. Additionally, *circDLGAP4* is found to relieve damage from ischemic stroke in brain tissue [82]. The ectopic expression of *circVMA21* decreases intervertebral disc degeneration of NP cells [83], while *circZNF609* regulates retinal neurodegeneration in retinal ganglion cells and vascular dysfunction in endothelial cells [84, 85].

### The mechanisms of circRNA functions

#### CircRNAs as miRNA sponge

The most prominent function of circRNAs is its action as a miRNA sponge to regulate target gene expression by inhibiting miRNA activity. One circRNA can regulate one or multiple miRNAs through multiple miRNA binding sites in the circular sequence. For example, the first identified functional circRNA, human *CDR1as*, has 74 miR-7 binding sites, 63 of which were found to be conserved in one other species. *CDR1as* is shown to be enriched in neural tissues, and knocking out *CDR1as* expression in mouse or zebrafish impairs midbrain development through miR-7 dysregulation [15, 71, 86]. In human cells, knockdown of *CDR1as* expression also dysregulates miR-7 expression and affects insulin secretion, cell proliferation and the pathobiology of myocardial infarction [42, 44, 70, 71, 73, 87–90]. The testis-specific circular *SRY* controls sex determination in mammals [5]. Circular *SRY* has 16 miR-138 binding sites and was shown to interact with miR-138 and AGO2 in HEK293 cells, suggesting that *SRY* acts as a miR-138 sponge [16]. *circHIPK3* has 18 miRNA binding sites for nine different miRNAs, among which the inhibition of miR-124 activity promotes cell proliferation in HCC and gallbladder cancer cells [48, 91, 92]. c*ircHIPK3* also targets miR-338-3p to regulate insulin secretion by β-cells [74]. It is not surprising that circRNA has been shown to regulate different downstream genes through different miRNAs. For example, *circITCH* sequesters miR-214 and miR-22-3p to promote ITCH and CBL expression, thereby regulating the WNT/β-catenin pathway [54, 55]. *circITCH* also increases PTEN and RASA1 expression (components of PI3K/AKT and MAPKERK pathways) by targeting miR-17/224 and miR-145, respectively [53, 93]. Interestingly, circRNA may even target different miRNAs to exert opposite functions in different cells. For example, *circZFR* targets miR-130a/107 to upregulate PTEN and inhibits gastric cancer cell proliferation, but targets miR-1261/4302/3619 to promote HCC proliferation [47, 52, 94, 95]. Many circRNAs have been shown to function through sponging miRNAs, and we have summarized the known instances in Table 1.

**Table 1:** circRNAs that function as miRNA sponges

*CircRNA*	Biological functions	miRNA	Targets	Cell type	Ref
*CDR1as*	Neural development Insulin secretion Myocardial infarction Promotes proliferation Anti-oncogenic Promotes proliferation Promotes proliferation/metastasis Osteoblastic differentiation	miR-7/− 671 miR-7 miR-7 miR-876-5p miR-7/−135a miR-7 miR-7 miR-7	Fos Pax6, Myrip PARP, SP1 MAGE-A P21 CCNE1, PIK3CD, EGFR HOXB13 GDF5	Neural tissue Islet cells Cardiomyocytes ESCC Bladder cancer NSCLC ESCC PDLSC	[15, 42, 44, 70, 71, 73, 87–90]
*SRY*	Sex-determining	miR-138		Testis	[16]
*circBIRC6*	Pluripotency maintenance	miR-34a/−145	NANOG, OCT4, SOX2	hESCs, iPSCs	[36]
*circHIPK3*	Promotes proliferation	miR-124/− 152/−193a/−29a/−29b/− 338/− 379/− 584/− 654	IL6R, DLX2	Cancer tissues	[41, 46, 48, 74, 91, 92, 114]
	Inhibits cancer progression β-cell function Promotes proliferation Promotes proliferation/migration Promotes proliferation/migration Promotes proliferation	miR-558 miR-124-3p/338-3p miR-30a-3p miR-124 miR-7 miR-124	HPSE Slc2a2, Akt1, Mtpn FZD4, WNT2, VEGF-C AQP3 FAK, IGF1R, EGFR ROCK1, CDK6	Bladder cancer β-cells Retinal endothelial cells HCC CRC Gallbladder cancer	
*circWDR77*	Promotes proliferation	miR-124	FGF2	VSMC	[43]
*circNT5E*	Promotes cancer progression	miR-422a	PIK3CA, NT5E	Glioblastoma	[45]
*circZFR*	Promotes cancer progression Promotes cancer progression Promotes cancer progression Inhibits cancer progression	miR-3619-5p miR-4302 miR-1261 miR-130a/−107	CTNNB1 ZNF121 C8orf4 PTEN	HCC Lung cancer PTC Gastric Cancer	[47, 52, 94, 95]
*circTCF25*	Promotes cancer progression	miR-103a-3p/− 107	CDK6	Bladder carcinoma	[49]
*Hsa_circ_0008039 (circPRKAR1B)*	Promote proliferation/migration	miR-432-5p	E2F3	Breast cancer cells	[51]
*circITCH*	Inhibits proliferation Inhibits cancer progression Inhibits cancer progression Inhibits cancer progression	miR-214 miR-17/− 224 miR-22-3p miR-145	ITCH/CTNNB1 P21, PTEN CBL/CTNNB1 RASA1	CRC Bladder cancer Papillary thyroid cancer Ovarian cancer	[53–55, 93]
*Hsa_circ_0002052* *(circPAPPA)*	Inhibits cancer progression	miR-1205	APC2	Osteosarcoma	[56]
*circMYLK*	Promotes cancer progression	miR-29a	LAMC, TRAF4	PC-a	[58]
*circRNA_0084043* *(circADAM9)*	Promotes cancer progression	miR-153-3p	SNAIL	melanoma	[59]
*circIRAK3*	Promote migration/invasion	miR-3607	FOXC1	Breast cancer cells	[60]
*circNASP*	Promotes cancer progression	miR-1253	FOXF1	Osteosarcoma	[61]
*circMAN2B2*	Promotes proliferation/migration	miR-1275	FOXK1	Lung cancer	[62]
*circSHKBP1*	Promotes angiogenesis	miR-544a/− 379	FOXP1, FOXP2	Endothelial cells	[63]
*circSMAD2*	Inhibits EMT	miR-629	TRIM33	HCC	[64]
*circFOXO3*	Inhibits cancer progression	miR-155	FOXO3	NSCLC	[65]
*circFGFR4*	Myoblast differentiation	miR-107	WNT3A	Bovine myoblast	[67]
*circSVIL*	Myoblast differentiation	miR-203	MEF2C, JUN	Chicken myoblast	[68]
*circZC3H4*	Macrophage activation	miR-212	ZC3H4	Alveolar macrophage	[75]
*circHIPK2*	Astrocyte activation ER stress	miR-124 miR-506-3p	SIGMAR1 SIGMAR1	Astrocyte HPF-a	[77, 115]
*circHECTD1*	Inhibits astrocyte activation	miR-142	TIPARP	Brain	[78]
*circGRB10*	Inhibits apoptosis	miR-328-5p	ERBB2	NP cells	[79]
*Hsa_circ_0043256 (circACACA)*	Induced apoptosis	miR-1252	ITCH	NSCLC	[80]
*circDLGAP4*	Ameliorates ischemic stroke	miR-143	HECTD1	Brain tissue	[82]
*circVMA21*	Against IDD	miR-200c	XIAP	NP cells	[83]
*circZNF609*	Retinal neurodegeneration Vascular dysfunction Myoblast differentiation	miR-615 miR-615 miR-194-5p	METRN MEF2A BCLAF1	RGC Vascular endothelial C2C12	[84, 85, 116]
*circPVT1*	Promotes proliferation	miR-497-5p	Aurka, Bub1, mKi67	HNSCC	[117]
*circMTO1*	Inhibits cancer progression	miR-9	P21	HCC	[118]
*circITGA7*	Inhibits proliferation/metastasis	miR-370-3p	NF1	CRC	[119]
*circACTA2*	VSMC contraction	miR-548f-5p	SMA	HASMC	[120]
*circCCDC66*	Promotes cancer progression	miR-33b/− 93/− 185	DNMT3B, MYC, EZH2,	CRC	[121]
*circFBLIM1*	Promotes cancer progression	miR-346	FBLIM1	HCC	[122]
*circATP2B1*	Promotes invasion	miR-204-3p	FN1	CCRCC	[123]
*circLARP4*	Inhibits proliferation/invasion	miR-424-5p	LATS1	Gastric cancer	[124]
*Hsa_circ_0000799 (circBPTF)*	Promotes cancer progression	miR-31-5p	RAB27A	Bladder cancer	[125]
*circRNA_000203 (circMYO9A)*	Promotes fibrosis	miR-26b-5p	Col1a2, Col3a1, SMA, CTGF	Cardiac fibroblast	[126]
*circRNA_8924 (circC1orf116)*	Promotes cancer progression	miR-518d-5p/− 519-5p	CBX8	Cervical cancer cells	[127]
*circRNA_008913 (circADAT1)*	Reduces carcinogenesis	miR-889	DAB2IP	HaCaT	[128]

Abbreviations: *CCRCC* (Clear Cell Renal Cell Carcinoma), *CRC* (Colorectal cancer), *ESCC* (Esophageal squamous cell carcinoma), *HASMC* (Human aortic smooth muscle cells), *HCC* (Hepatocellular carcinoma), *HNSCC* (Head and neck squamous cell carcinoma), *IDD* (intervertebral disc degeneration), *NP* cells (Nucleus pulposus cells), *NSCLC* (Non-small-cell lung carcinoma), *PDLSC* (Periodontal ligament stem cells), *PTC* (Papillary thyroid cancer), *RGC* (Retinal ganglion cells), *VSMC* (Vascular smooth muscle cells)

#### CircRNAs as protein decoys

In addition to interacting with miRNAs, circRNAs can serve as protein decoys to influence cellular functions. For example, *circFOXO3* is shown to trap CDK2/p21 and HIF-a/ID1 in the cytoplasm, which blocks cell cycle progression and induces cell senescence, respectively [23, 96]. *circFOXO3* also promotes the interaction between MDM2 and P53, which decreases the P53 protein level and induces apoptosis [97]. In breast cancer cells, *circDNMT1* activates autophagy by promoting P53 and AUF1 nuclear translocation [98]. In vascular tissue, *circANRIL* sequesters PES1 to impair rRNA maturation, resulting in apoptosis [81]. In glioblastoma multiforme cells, *circSMARCA5* inhibited migration by stimulating splicing factor SRSF1 to modulate expression of the SRSF3 isoform [99]. In breast cancer cells, *circMTO1* sequesters TRAF4, preventing Eg5 activation and decreasing cell viability [100]. In primary cardiomyocytes, *circAmotl1* interacts with PDK1 and AKT1, which induced the phosphorylation and nuclear translocation of AKT1, reducing apoptosis to promote cardiac repair [101]. In HeLa cells, *circPABPN1* recruits HuR to suppress its interaction with PABPN1 mRNA, which led to reduced PABPN1 translation [24]. These protein decoy functions of circRNAs are summarized in Table 2.

**Table 2:** CircRNAs that function as protein decoys

*CircRNA*	Biological functions	Interacting protein	Cell type	Ref
*circFOXO3*	Inhibits cell cycle progression Cardiac senescence Induces apoptosis	P21, CDK2 ID-1, E2F1, FAK, HIF1α MDM2, P53	Non-cancer cells Heart tissue Non-cancer cells	[96, 97, 129]
*circANRIL*	rRNA maturation	PES1	Vascular tissue	[81]
*circHECTD1*	Macrophage activation	ZC3H12A	Macrophage	[76]
*circDNMT1*	Promotes proliferation	P53, AUF1	Breast cancer cells	[98]
*circSMARCA5*	Tumor suppressor	SRSF1	Glioblastoma	[99]
*circMTO1*	Inhibits proliferation	TRAF4	Breast cancer cells	[100]
*circAMOTL1*	Promotes cell survival	PDK1, AKT1	Cardiomyocytes	[101]
*circPABPN1*	Suppresses PABPN1 translation	HuR	HeLa	[24]

#### Translatable circRNAs

Although circRNAs are considered to be lncRNAs with low protein coding potential, it has been shown that circRNAs containing an internal ribosome entry site (IRES) or N^6^-methyladenosine modification and can be translated into peptides in vitro and in vivo [28, 102–105]. Notably, many circRNAs contain the start codon of cognate mRNAs associated with ribosomes [29]. These findings indicate that circRNAs are sometimes able to be translated. Pamudurti et al. further shows that endogenous *circMbl3* produces a detectable protein product in fly head by targeted mass spectrometry analysis of Mbl immunoprecipitate [29]. Importantly, Legnini et al. demonstrates that *circZNF609* regulates myogenesis and can be translated into peptides, suggesting that *circZNF609* may exert its function through protein expression [27]. Unfortunately, the phenotype could not be unequivocally linked to protein products because the re-expression of *circZNF609* by plasmids or naked RNA induces a non-specific block of myoblast proliferation. In addition, Zhang et al. finds that circular *lncRNA-PINT* can be translated into a small peptide to suppress glioblastoma cell proliferation; this action is mediated by trapping of PAF1c to inhibit translational elongation of oncogenes [30]. Moreover, some specific circRNAs are found to be associated with translating ribosomes in mammalian cells [29], which is highly suggestive that these circRNAs produce functional peptides.

### The biogenesis of CircRNAs

CircRNAs are generated by back-splicing, wherein the 3′ terminus of a downstream exon is ligated to the 5′ terminus of an upstream exon. Similar to canonical splicing, back-splicing of circRNAs is tightly regulated by *cis*-elements (i.e., DNA sequences) and trans-factors (i.e., RNA binding proteins). Generally, most circRNAs contain two or three exons without intron segregation, while those circRNAs that contain only one exon typically exhibit a longer than average exon length [35]. Nevertheless, analysis of circular exon sequences and circular exon replacement assays both suggest that there are no specific exonic sequences that control circRNA formation [32]. On the other hand, the flanking introns of circRNAs are usually longer than average and enriched with complementary repeats [12, 35, 106]. Capel et al. are the first to show that complementary intronic sequences (CIS) flanked the circular *SRY* gene in mouse, suggesting that CIS may mediate the formation of this circRNA [5]. Further studies indicated that CIS are enriched in flanking introns of circRNAs from various species, including mouse, pig, *C. elegans* and *Drosophila* [32, 106–108]. Importantly, deletion of CIS adjacent to Laccase2 exon 2 abolishes circular laccase2 expression in *Drosophila* [38]*.* Furthermore, the primate-specific Alu repetitive elements, have been implicated in the biogenesis of some circRNAs. Jeck et al. first demonstrates that Alu repetitive elements are enriched in the flanking introns of human circRNAs [12], and Zhang et al. extends this observation, confirming that the pairing between Alu repetitive elements with reverse orientation regulates the expression of linear and circular isoforms [35, 109].

With regard to trans-factors in circRNA formation, Ashwal-Fluss et al. showed that the Mbl binding sites on flanking introns are necessary for circMbl formation; furthermore, ectopic expression of Mbl enhances circMbl expression, suggesting that the splicing factor was involved in circRNA biogenesis [32]. Conn et al. further demonstrates that the disruption of splicing factor QKI or its binding sites on flanking introns attenuates circRNA formation during EMT, and Errichelli et al. find that disruption of splicing factor FUS in mouse motor neurons affects circRNA expression [110]. Our group also show that splicing factor ESRP1 can promote circRNA expression through intronic binding sites flanking *circBIRC6* in human ESCs [36]. In addition to promoting circRNA biogenesis, splicing factors have also been shown to repress circRNA formation. For example, disruption of SR family members SRSF1/6/11 or hnRNP family member Hrb27C enhances circular laccase2 expression in *Drosophila* [38]. In addition, double-stranded RNA binding proteins, such as ILF3 (NF90/NF110) or DHX9, also have been shown to regulate circRNA formation. Disruption of ILF3 (NF90/NF110) downregulates circRNA expression, while disruption of DHX9 upregulates circRNA expression in human cells [111, 112]. The binding of ILF3 (NF90/NF110) is shown to stabilize CIS pairs, while the binding of DHX9 recruits ADAR1 to disrupt the pairing of Alu repetitive elements through A to I editing.

## Conclusion

In this review, we survey the known functions of circRNAs in cell proliferation, EMT, development and other cellular processes. We also summarize the mechanisms by which circRNAs function, including RNA and protein interactions, and we describe the regulatory elements that are known to be involved in circRNA formation. Despite the broad range of findings regarding circRNA functions and regulation, many questions remain to be resolved. For example, how circRNAs are degraded in the cell and how degradation works in conjunction with biogenesis to respond to dynamic cellular states is an important territory that awaits further exploration. Some researchers have suggested that exocytosis may be an important pathway for circRNA clearance [113], but the selective enrichment of circRNAs in exosomes from different cell types argues against to this model [26]. Although the expression of circRNAs has been studied in the context of many human diseases, our understanding of the different roles in normal physiology and the disease conditions is limited for the vast majority of identified circRNAs. Finally, improvements in technology to detect circRNAs at a single-cell level and methods to efficiently manipulate circRNAs without affecting linear cognates will be key for gaining further insights into the functions of circRNAs and the mechanisms underpinning their regulatory roles.

## Abbreviations

CCRCC: Clear Cell Renal Cell Carcinoma
CircRNAs: Circular RNA
CIS: Complementary intronic sequences
CRC: Colorectal cancer
EMT: Epithelial-mesenchymal transition
ESCC: Esophageal squamous cell carcinoma
HASMC: Human aortic smooth muscle cells
HCC: Hepatocellular carcinoma
HNSCC: Head and neck squamous cell carcinoma
IDD: Intervertebral disc degeneration
IRES: Internal ribosome entry site
LncRNAs: Long non-coding RNAs
miRNAs: micro RNAs
NP cells: Nucleus pulposus cells
NSCLC: Non-small-cell lung carcinoma
PDLSC: Periodontal ligament stem cells
PTC: Papillary thyroid cancer
RGC: Retinal ganglion cells
VSMC: Vascular smooth muscle cells

## References

[1] Braunschweig U, Gueroussov S, Plocik AM, Graveley BR, Blencowe BJ (2013). Dynamic integration of splicing within gene regulatory pathways. Cell..

[2] Wang ET, Sandberg R, Luo S, Khrebtukova I, Zhang L, Mayr C (2008). Alternative isoform regulation in human tissue transcriptomes. Nature..

[3] Enuka Y, Lauriola M, Feldman ME, Sas-Chen A, Ulitsky I, Yarden Y (2016). Circular RNAs are long-lived and display only minimal early alterations in response to a growth factor. Nucleic Acids Res.

[4] Hsu MT, Coca-Prados M (1979). Electron microscopic evidence for the circular form of RNA in the cytoplasm of eukaryotic cells. Nature..

[5] Capel B, Swain A, Nicolis S, Hacker A, Walter M, Koopman P (1993). Circular transcripts of the testis-determining gene Sry in adult mouse testis. Cell..

[6] Cocquerelle C, Daubersies P, Majerus MA, Kerckaert JP, Bailleul B (1992). Splicing with inverted order of exons occurs proximal to large introns. EMBO J.

[7] Nigro JM, Cho KR, Fearon ER, Kern SE, Ruppert JM, Oliner JD (1991). Scrambled exons. Cell..

[8] Zaphiropoulos PG (1996). Circular RNAs from transcripts of the rat cytochrome P450 2C24 gene: correlation with exon skipping. Proc Natl Acad Sci U S A.

[9] Zaphiropoulos PG (1997). Exon skipping and circular RNA formation in transcripts of the human cytochrome P-450 2C18 gene in epidermis and of the rat androgen binding protein gene in testis. Mol Cell Biol.

[10] Rybak-Wolf A, Stottmeister C, Glazar P, Jens M, Pino N, Giusti S (2015). Circular RNAs in the mammalian brain are highly abundant, conserved, and dynamically expressed. Mol Cell.

[11] Salzman J, Chen RE, Olsen MN, Wang PL, Brown PO (2013). Cell-type specific features of circular RNA expression. PLoS Genet.

[12] Jeck WR, Sorrentino JA, Wang K, Slevin MK, Burd CE, Liu J (2013). Circular RNAs are abundant, conserved, and associated with ALU repeats. RNA..

[13] Salzman J, Gawad C, Wang PL, Lacayo N, Brown PO (2012). Circular RNAs are the predominant transcript isoform from hundreds of human genes in diverse cell types. PLoS One.

[14] Guo JU, Agarwal V, Guo H, Bartel DP (2014). Expanded identification and characterization of mammalian circular RNAs. Genome Biol.

[15] Memczak S, Jens M, Elefsinioti A, Torti F, Krueger J, Rybak A (2013). Circular RNAs are a large class of animal RNAs with regulatory potency. Nature..

[16] Hansen TB, Jensen TI, Clausen BH, Bramsen JB, Finsen B, Damgaard CK (2013). Natural RNA circles function as efficient microRNA sponges. Nature..

[17] Xia S, Feng J, Chen K, Ma Y, Gong J, Cai F (2018). CSCD: a database for cancer-specific circular RNAs. Nucleic Acids Res.

[18] Glazar P, Papavasileiou P, Rajewsky N (2014). circBase: a database for circular RNAs. RNA..

[19] Ghosal S, Das S, Sen R, Basak P, Chakrabarti J (2013). Circ2Traits: a comprehensive database for circular RNA potentially associated with disease and traits. Front Genet.

[20] Liu YC, Li JR, Sun CH, Andrews E, Chao RF, Lin FM (2016). CircNet: a database of circular RNAs derived from transcriptome sequencing data. Nucleic Acids Res.

[21] Yao D, Zhang L, Zheng M, Sun X, Lu Y, Liu P (2018). Circ2Disease: a manually curated database of experimentally validated circRNAs in human disease. Sci Rep.

[22] Li S, Li Y, Chen B, Zhao J, Yu S, Tang Y (2018). exoRBase: a database of circRNA, lncRNA and mRNA in human blood exosomes. Nucleic Acids Res.

[23] Du WW, Yang W, Liu E, Yang Z, Dhaliwal P, Yang BB. Foxo3 circular RNA retards cell cycle progression via forming ternary complexes with p21 and CDK2. Nucleic Acids Res. 2016.10.1093/nar/gkw027PMC482410426861625

[24] Abdelmohsen K, Panda AC, Munk R, Grammatikakis I, Dudekula DB, De S (2017). Identification of HuR target circular RNAs uncovers suppression of PABPN1 translation by CircPABPN1. RNA Biol.

[25] Zhao RT, Zhou J (2018). Dong XL.

[26] Preusser C, Hung LH, Schneider T, Schreiner S, Hardt M, Moebus A (2018). Selective release of circRNAs in platelet-derived extracellular vesicles. J Extracell Vesicles.

[27] Legnini I, Di Timoteo G, Rossi F, Morlando M, Briganti F, Sthandier O (2017). Circ-ZNF609 is a circular RNA that can be translated and functions in Myogenesis. Mol Cell.

[28] Wang Y, Wang Z (2015). Efficient backsplicing produces translatable circular mRNAs. RNA..

[29] Pamudurti NR, Bartok O, Jens M, Ashwal-Fluss R, Stottmeister C, Ruhe L (2017). Translation of CircRNAs. Mol Cell.

[30] Zhang M, Zhao K, Xu X, Yang Y, Yan S, Wei P (2018). A peptide encoded by circular form of LINC-PINT suppresses oncogenic transcriptional elongation in glioblastoma. Nat Commun.

[31] Starke S, Jost I, Rossbach O, Schneider T, Schreiner S, Hung LH (2015). Exon circularization requires canonical splice signals. Cell Rep.

[32] Ashwal-Fluss R, Meyer M, Pamudurti NR, Ivanov A, Bartok O, Hanan M (2014). circRNA biogenesis competes with pre-mRNA splicing. Mol Cell.

[33] Liang D, Wilusz JE (2014). Short intronic repeat sequences facilitate circular RNA production. Genes Dev.

[34] Ivanov A, Memczak S, Wyler E, Torti F, Porath HT, Orejuela MR (2015). Analysis of intron sequences reveals hallmarks of circular RNA biogenesis in animals. Cell Rep.

[35] Zhang XO, Wang HB, Zhang Y, Lu X, Chen LL, Yang L (2014). Complementary sequence-mediated exon circularization. Cell..

[36] Yu CY, Li TC, Wu YY, Yeh CH, Chiang W, Chuang CY (2017). The circular RNA circBIRC6 participates in the molecular circuitry controlling human pluripotency. Nat Commun.

[37] Conn SJ, Pillman KA, Toubia J, Conn VM, Salmanidis M, Phillips CA (2015). The RNA binding protein quaking regulates formation of circRNAs. Cell..

[38] Kramer MC, Liang D, Tatomer DC, Gold B, March ZM, Cherry S (2015). Combinatorial control of Drosophila circular RNA expression by intronic repeats, hnRNPs, and SR proteins. Genes Dev.

[39] Homem CC, Repic M, Knoblich JA (2015). Proliferation control in neural stem and progenitor cells. Nat Rev Neurosci.

[40] Kastan MB, Bartek J (2004). Cell-cycle checkpoints and cancer. Nature..

[41] Zeng K, Chen X, Xu M, Liu X, Hu X, Xu T (2018). CircHIPK3 promotes colorectal cancer growth and metastasis by sponging miR-7. Cell Death Dis.

[42] Li RC, Ke S, Meng FK, Lu J, Zou XJ, He ZG (2018). CiRS-7 promotes growth and metastasis of esophageal squamous cell carcinoma via regulation of miR-7/HOXB13. Cell Death Dis.

[43] Chen J, Cui L, Yuan J, Zhang Y, Sang H (2017). Circular RNA WDR77 target FGF-2 to regulate vascular smooth muscle cells proliferation and migration by sponging miR-124. Biochem Biophys Res Commun.

[44] Yu L, Gong X, Sun L, Zhou Q, Lu B, Zhu L (2016). The circular RNA Cdr1as act as an oncogene in hepatocellular carcinoma through targeting miR-7 expression. PLoS One.

[45] Wang R, Zhang S, Chen X, Li N, Li J, Jia R, et al. CircNT5E acts as a sponge of microRNA-422a to promote glioblastoma tumorigenesis. Cancer Res. 2018.10.1158/0008-5472.CAN-18-053229967262

[46] Shan K, Liu C, Liu BH, Chen X, Dong R, Liu X (2017). Circular noncoding RNA HIPK3 mediates retinal vascular dysfunction in diabetes mellitus. Circulation..

[47] Tan A, Li Q, Chen L (2018). CircZFR promotes hepatocellular carcinoma progression through regulating miR-3619-5p/CTNNB1 axis and activating Wnt/beta-catenin pathway. Arch Biochem Biophys.

[48] Zheng Q, Bao C, Guo W, Li S, Chen J, Chen B (2016). Circular RNA profiling reveals an abundant circHIPK3 that regulates cell growth by sponging multiple miRNAs. Nat Commun.

[49] Zhong Z, Lv M, Chen J (2016). Screening differential circular RNA expression profiles reveals the regulatory role of circTCF25-miR-103a-3p/miR-107-CDK6 pathway in bladder carcinoma. Sci Rep.

[50] Chen L, Zhang S, Wu J, Cui J, Zhong L, Zeng L (2017). circRNA_100290 plays a role in oral cancer by functioning as a sponge of the miR-29 family. Oncogene..

[51] Liu Y, Lu C, Zhou Y, Zhang Z, Sun L (2018). Circular RNA hsa_circ_0008039 promotes breast cancer cell proliferation and migration by regulating miR-432-5p/E2F3 axis. Biochem Biophys Res Commun.

[52] Liu T, Liu S, Xu Y, Shu R, Wang F, Chen C, et al. Circular RNA-ZFR inhibited cell proliferation and promoted apoptosis in gastric Cancer by sponging miR-130a/miR-107 and modulating PTEN. Cancer Res Treat. 2018.10.4143/crt.2017.537PMC619292429361817

[53] Yang C, Yuan W, Yang X, Li P, Wang J, Han J (2018). Circular RNA circ-ITCH inhibits bladder cancer progression by sponging miR-17/miR-224 and regulating p21. PTEN expression Mol Cancer.

[54] Huang Guanli, Zhu Hua, Shi Yixiong, Wu Wenzhi, Cai Huajie, Chen Xiangjian (2015). cir-ITCH Plays an Inhibitory Role in Colorectal Cancer by Regulating the Wnt/β-Catenin Pathway. PLOS ONE.

[55] Wang M, Chen B, Ru Z, Cong L (2018). CircRNA circ-ITCH suppresses papillary thyroid cancer progression through miR-22-3p/CBL/beta-catenin pathway. Biochem Biophys Res Commun.

[56] Wu Z, Shi W, Jiang C (2018). Overexpressing circular RNA hsa_circ_0002052 impairs osteosarcoma progression via inhibiting Wnt/beta-catenin pathway by regulating miR-1205/APC2 axis. Biochem Biophys Res Commun.

[57] Lamouille S, Xu J, Derynck R (2014). Molecular mechanisms of epithelial-mesenchymal transition. Nat Rev Mol Cell Biol.

[58] Dai Y, Li D, Chen X, Tan X, Gu J, Chen M (2018). Circular RNA myosin light chain kinase (MYLK) promotes prostate Cancer progression through modulating Mir-29a expression. Med Sci Monit.

[59] Luan W, Shi Y, Zhou Z, Xia Y, Wang J (2018). circRNA_0084043 promote malignant melanoma progression via miR-153-3p/Snail axis. Biochem Biophys Res Commun.

[60] Wu J, Jiang Z, Chen C, Hu Q, Fu Z, Chen J (2018). CircIRAK3 sponges miR-3607 to facilitate breast cancer metastasis. Cancer Lett.

[61] Huang L, Chen M, Pan J, Yu W (2018). Circular RNA circNASP modulates the malignant behaviors in osteosarcoma via miR-1253/FOXF1 pathway. Biochem Biophys Res Commun.

[62] Ma X, Yang X, Bao W, Li S, Liang S, Sun Y (2018). Circular RNA circMAN2B2 facilitates lung cancer cell proliferation and invasion via miR-1275/FOXK1 axis. Biochem Biophys Res Commun.

[63] He Qianru, Zhao Lini, Liu Yunhui, Liu Xiaobai, Zheng Jian, Yu Hai, Cai Heng, Ma Jun, Liu Libo, Wang Ping, Li Zhen, Xue Yixue (2018). circ-SHKBP1 Regulates the Angiogenesis of U87 Glioma-Exposed Endothelial Cells through miR-544a/FOXP1 and miR-379/FOXP2 Pathways. Molecular Therapy - Nucleic Acids.

[64] Zhang X, Luo P, Jing W, Zhou H, Liang C, Tu J (2018). circSMAD2 inhibits the epithelial-mesenchymal transition by targeting miR-629 in hepatocellular carcinoma. Onco Targets Ther.

[65] Zhang Y, Zhao H, Zhang L (2018). Identification of the tumorsuppressive function of circular RNA FOXO3 in nonsmall cell lung cancer through sponging miR155. Mol Med Rep.

[66] Izuogu OG, Alhasan AA, Mellough C, Collin J, Gallon R, Hyslop J (2018). Analysis of human ES cell differentiation establishes that the dominant isoforms of the lncRNAs RMST and FIRRE are circular. BMC Genomics.

[67] Li H, Wei X, Yang J, Dong D, Hao D, Huang Y (2018). circFGFR4 promotes differentiation of myoblasts via binding miR-107 to relieve its inhibition of Wnt3a. Mol Ther Nucleic Acids.

[68] Ouyang H, Chen X, Li W, Li Z, Nie Q, Zhang X (2018). Circular RNA circSVIL promotes myoblast proliferation and differentiation by sponging miR-203 in chicken. Front Genet.

[69] Wang Y, Li M, Wang Y, Liu J, Zhang M, Fang X (2019). A Zfp609 circular RNA regulates myoblast differentiation by sponging miR-194-5p. Int J Biol Macromol.

[70] Li X, Zheng Y, Zheng Y, Huang Y, Zhang Y, Jia L (2018). Circular RNA CDR1as regulates osteoblastic differentiation of periodontal ligament stem cells via the miR-7/GDF5/SMAD and p38 MAPK signaling pathway. Stem Cell Res Ther.

[71] Piwecka Monika, Glažar Petar, Hernandez-Miranda Luis R., Memczak Sebastian, Wolf Susanne A., Rybak-Wolf Agnieszka, Filipchyk Andrei, Klironomos Filippos, Cerda Jara Cledi Alicia, Fenske Pascal, Trimbuch Thorsten, Zywitza Vera, Plass Mireya, Schreyer Luisa, Ayoub Salah, Kocks Christine, Kühn Ralf, Rosenmund Christian, Birchmeier Carmen, Rajewsky Nikolaus (2017). Loss of a mammalian circular RNA locus causes miRNA deregulation and affects brain function. Science.

[72] Berta P, Hawkins JR, Sinclair AH, Taylor A, Griffiths BL, Goodfellow PN (1990). Genetic evidence equating SRY and the testis-determining factor. Nature..

[73] Xu H, Guo S, Li W, Yu P (2015). The circular RNA Cdr1as, via miR-7 and its targets, regulates insulin transcription and secretion in islet cells. Sci Rep.

[74] Stoll L, Sobel J, Rodriguez-Trejo A, Guay C, Lee K, Veno MT (2018). Circular RNAs as novel regulators of beta-cell functions in normal and disease conditions. Mol Metab.

[75] Yang X, Wang J, Zhou Z, Jiang R, Huang J, Chen L (2018). Silica-induced initiation of circular ZC3H4 RNA/ZC3H4 pathway promotes the pulmonary macrophage activation. FASEB J.

[76] Zhou Z, Jiang R, Yang X, Guo H, Fang S, Zhang Y (2018). circRNA mediates silica-induced macrophage activation via HECTD1/ZC3H12A-dependent ubiquitination. Theranostics..

[77] Huang R, Zhang Y, Han B, Bai Y, Zhou R, Gan G (2017). Circular RNA HIPK2 regulates astrocyte activation via cooperation of autophagy and ER stress by targeting MIR124-2HG. Autophagy..

[78] Han B, Zhang Y, Zhang Y, Bai Y, Chen X, Huang R, et al. Novel insight into circular RNA HECTD1 in astrocyte activation via autophagy by targeting MIR142-TIPARP: implications for cerebral ischemic stroke. Autophagy. 2018:1–21.10.1080/15548627.2018.1458173PMC610366029938598

[79] Guo W, Zhang B, Mu K, Feng SQ, Dong ZY, Ning GZ (2018). Circular RNA GRB10 as a competitive endogenous RNA regulating nucleus pulposus cells death in degenerative intervertebral disk. Cell Death Dis.

[80] Tian F, Yu CT, Ye WD, Wang Q (2017). Cinnamaldehyde induces cell apoptosis mediated by a novel circular RNA hsa_circ_0043256 in non-small cell lung cancer. Biochem Biophys Res Commun.

[81] Holdt LM, Stahringer A, Sass K, Pichler G, Kulak NA, Wilfert W (2016). Circular non-coding RNA ANRIL modulates ribosomal RNA maturation and atherosclerosis in humans. Nat Commun.

[82] Bai Y, Zhang Y, Han B, Yang L, Chen X, Huang R (2018). Circular RNA DLGAP4 ameliorates ischemic stroke outcomes by targeting miR-143 to regulate endothelial-mesenchymal transition associated with blood-brain barrier integrity. J Neurosci.

[83] Cheng X, Zhang L, Zhang K, Zhang G, Hu Y, Sun X (2018). Circular RNA VMA21 protects against intervertebral disc degeneration through targeting miR-200c and X linked inhibitor-of-apoptosis protein. Ann Rheum Dis.

[84] Liu C, Yao MD, Li CP, Shan K, Yang H, Wang JJ (2017). Silencing of circular RNA-ZNF609 ameliorates vascular endothelial dysfunction. Theranostics..

[85] Wang JJ, Liu C, Shan K, Liu BH, Li XM, Zhang SJ (2018). Circular RNA-ZNF609 regulates retinal neurodegeneration by acting as miR-615 sponge. Theranostics..

[86] Kleaveland B, Shi CY, Stefano J, Bartel DP (2018). A network of noncoding regulatory RNAs acts in the mammalian brain. Cell..

[87] Li P, Yang X, Yuan W, Yang C, Zhang X, Han J (2018). CircRNA-Cdr1as exerts anti-oncogenic functions in bladder Cancer by sponging MicroRNA-135a. Cell Physiol Biochem.

[88] Geng HH, Li R, Su YM, Xiao J, Pan M, Cai XX (2016). The circular RNA Cdr1as promotes myocardial infarction by mediating the regulation of miR-7a on its target genes expression. PLoS One.

[89] Zhang X, Yang D, Wei Y (2018). Overexpressed CDR1as functions as an oncogene to promote the tumor progression via miR-7 in non-small-cell lung cancer. Onco Targets Ther..

[90] Sang M, Meng L, Sang Y, Liu S, Ding P, Ju Y (2018). Circular RNA ciRS-7 accelerates ESCC progression through acting as a miR-876-5p sponge to enhance MAGE-A family expression. Cancer Lett.

[91] Chen G, Shi Y, Liu M, Sun J. circHIPK3 regulates cell proliferation and migration by sponging miR-124 and regulating AQP3 expression in hepatocellular carcinoma. Cell Death Dis. 2018;9(2):175.10.1038/s41419-017-0204-3PMC583372429415990

[92] Kai D, Yannian L, Yitian C, Dinghao G, Xin Z, Wu J. Circular RNA HIPK3 promotes gallbladder cancer cell growth by sponging microRNA-124. Biochem Biophys Res Commun. 2018.10.1016/j.bbrc.2018.06.08829928876

[93] Hu J, Wang L, Chen J, Gao H, Zhao W, Huang Y, et al. The circular RNA circ-ITCH suppresses ovarian carcinoma progression through targeting miR-145/RASA1 signaling. Biochem Biophys Res Commun. 2018.10.1016/j.bbrc.2018.09.06030243714

[94] Wei H, Pan L, Tao D, Li R (2018). Circular RNA circZFR contributes to papillary thyroid cancer cell proliferation and invasion by sponging miR-1261 and facilitating C8orf4 expression. Biochem Biophys Res Commun.

[95] Liu W, Ma W, Yuan Y, Zhang Y, Sun S (2018). Circular RNA hsa_circRNA_103809 promotes lung cancer progression via facilitating ZNF121-dependent MYC expression by sequestering miR-4302. Biochem Biophys Res Commun.

[96] Du WW, Yang W, Chen Y, Wu ZK, Foster FS, Yang Z (2017). Foxo3 circular RNA promotes cardiac senescence by modulating multiple factors associated with stress and senescence responses. Eur Heart J.

[97] Du WW, Fang L, Yang W, Wu N, Awan FM, Yang Z (2017). Induction of tumor apoptosis through a circular RNA enhancing Foxo3 activity. Cell Death Differ.

[98] Du WW, Yang W, Li X, Awan FM, Yang Z, Fang L, et al. A circular RNA circ-DNMT1 enhances breast cancer progression by activating autophagy. Oncogene. 2018.10.1038/s41388-018-0369-y29973691

[99] Barbagallo Davide, Caponnetto Angela, Cirnigliaro Matilde, Brex Duilia, Barbagallo Cristina, D’Angeli Floriana, Morrone Antonio, Caltabiano Rosario, Barbagallo Giuseppe, Ragusa Marco, Di Pietro Cinzia, Hansen Thomas, Purrello Michele (2018). CircSMARCA5 Inhibits Migration of Glioblastoma Multiforme Cells by Regulating a Molecular Axis Involving Splicing Factors SRSF1/SRSF3/PTB. International Journal of Molecular Sciences.

[100] Liu Y, Dong Y, Zhao L, Su L, Luo J (2018). Circular RNAMTO1 suppresses breast cancer cell viability and reverses monastrol resistance through regulating the TRAF4/Eg5 axis. Int J Oncol.

[101] Zeng Y, Du WW, Wu Y, Yang Z, Awan FM, Li X (2017). A circular RNA binds to and activates AKT phosphorylation and nuclear localization reducing apoptosis and enhancing cardiac repair. Theranostics..

[102] Abe N, Matsumoto K, Nishihara M, Nakano Y, Shibata A, Maruyama H (2015). Rolling circle translation of circular RNA in living human cells. Sci Rep.

[103] Chen CY, Sarnow P (1995). Initiation of protein synthesis by the eukaryotic translational apparatus on circular RNAs. Science..

[104] Yang Y, Fan X, Mao M, Song X, Wu P, Zhang Y (2017). Extensive translation of circular RNAs driven by N(6)-methyladenosine. Cell Res.

[105] Wesselhoeft RA, Kowalski PS, Anderson DG (2018). Engineering circular RNA for potent and stable translation in eukaryotic cells. Nat Commun.

[106] Westholm JO, Miura P, Olson S, Shenker S, Joseph B, Sanfilippo P (2014). Genome-wide analysis of drosophila circular RNAs reveals their structural and sequence properties and age-dependent neural accumulation. Cell Rep.

[107] Barrett SP, Wang PL, Salzman J (2015). Circular RNA biogenesis can proceed through an exon-containing lariat precursor. Elife..

[108] Kristensen LS, Okholm TLH, Veno MT, Kjems J (2018). Circular RNAs are abundantly expressed and upregulated during human epidermal stem cell differentiation. RNA Biol.

[109] Zhang Y, Xue W, Li X, Zhang J, Chen S, Zhang JL (2016). The biogenesis of nascent circular RNAs. Cell Rep.

[110] Errichelli L, Dini Modigliani S, Laneve P, Colantoni A, Legnini I, Capauto D (2017). FUS affects circular RNA expression in murine embryonic stem cell-derived motor neurons. Nat Commun.

[111] Li X, Liu CX, Xue W, Zhang Y, Jiang S, Yin QF (2017). Coordinated circRNA biogenesis and function with NF90/NF110 in viral infection. Mol Cell.

[112] Aktas T, Avsar Ilik I, Maticzka D, Bhardwaj V, Pessoa Rodrigues C, Mittler G (2017). DHX9 suppresses RNA processing defects originating from the Alu invasion of the human genome. Nature..

[113] Lasda E, Parker R (2016). Circular RNAs co-precipitate with extracellular vesicles: a possible mechanism for circRNA clearance. PLoS One.

[114] Li Y, Zheng F, Xiao X, Xie F, Tao D, Huang C (2017). CircHIPK3 sponges miR-558 to suppress heparanase expression in bladder cancer cells. EMBO Rep.

[115] Cao Z, Xiao Q, Dai X, Zhou Z, Jiang R, Cheng Y, et al. circHIPK2-mediated sigma-1R promotes endoplasmic reticulum stress in human pulmonary fibroblasts exposed to silica. Cell Death Dis. 2017;8(12):3212.10.1038/s41419-017-0017-4PMC587058729238093

[116] Wang Y, Li M, Wang Y, Liu J, Zhang M, Fang X, et al. A Zfp609 circular RNA regulates myoblast differentiation by sponging miR-194-5p. Int J Biol Macromol. 2018.10.1016/j.ijbiomac.2018.09.03930201567

[117] Verduci L, Ferraiuolo M, Sacconi A, Ganci F, Vitale J, Colombo T (2017). The oncogenic role of circPVT1 in head and neck squamous cell carcinoma is mediated through the mutant p53/YAP/TEAD transcription-competent complex. Genome Biol.

[118] Han D, Li J, Wang H, Su X, Hou J, Gu Y (2017). Circular RNA circMTO1 acts as the sponge of microRNA-9 to suppress hepatocellular carcinoma progression. Hepatology..

[119] Li X, Wang J, Zhang C, Lin C, Zhang J, Zhang W, et al. Circular RNA circITGA7 inhibits colorectal cancer growth and metastasis by modulating the Ras pathway and upregulating transcription of its host gene ITGA7. J Pathol. 2018.10.1002/path.512529943828

[120] Sun Y, Yang Z, Zheng B, Zhang XH, Zhang ML, Zhao XS (2017). A novel regulatory mechanism of smooth muscle alpha-actin expression by NRG-1/circACTA2/miR-548f-5p Axis. Circ Res.

[121] Hsiao KY, Lin YC, Gupta SK, Chang N, Yen L, Sun HS (2017). Noncoding effects of circular RNA CCDC66 promote Colon Cancer growth and metastasis. Cancer Res.

[122] Bai N, Peng E, Qiu X, Lyu N, Zhang Z, Tao Y, et al. circFBLIM1 act as a ceRNA to promote hepatocellular cancer progression by sponging miR-346. J Exp Clin Cancer Res. 2018;37(1):172.10.1186/s13046-018-0838-8PMC606299130053867

[123] Han Z, Zhang Y, Sun Y, Chen J, Chang C, Wang X (2018). ERbeta-mediated alteration of circATP2B1 and miR-204-3p signaling promotes invasion of clear cell renal cell carcinoma. Cancer Res.

[124] Zhang J, Liu H, Hou L, Wang G, Zhang R, Huang Y (2017). Circular RNA_LARP4 inhibits cell proliferation and invasion of gastric cancer by sponging miR-424-5p and regulating LATS1 expression. Mol Cancer.

[125] Bi J, Liu H, Cai Z, Dong W, Jiang N, Yang M, et al. Circ-BPTF promotes bladder cancer progression and recurrence through the miR-31-5p/RAB27A axis. Aging (Albany NY). 2018.10.18632/aging.101520PMC612844030103209

[126] Tang CM, Zhang M, Huang L, Hu ZQ, Zhu JN, Xiao Z (2017). CircRNA_000203 enhances the expression of fibrosis-associated genes by derepressing targets of miR-26b-5p, Col1a2 and CTGF, in cardiac fibroblasts. Sci Rep.

[127] Liu J, Wang D, Long Z, Liu J, Li W (2018). CircRNA8924 promotes cervical Cancer cell proliferation, migration and invasion by competitively binding to MiR-518d-5p /519-5p family and modulating the expression of CBX8. Cell Physiol Biochem.

[128] Xiao T, Xue J, Shi M, Chen C, Luo F, Xu H, et al. Circ008913, via miR-889 regulation of DAB2IP/ZEB1, is involved in the arsenite-induced acquisition of CSC-like properties by human keratinocytes in carcinogenesis. Metallomics. 2018.10.1039/c8mt00207j30167605

[129] Du WW, Yang W, Liu E, Yang Z, Dhaliwal P, Yang BB (2016). Foxo3 circular RNA retards cell cycle progression via forming ternary complexes with p21 and CDK2. Nucleic Acids Res.

